# Intelligent Recognition Model of Business English Translation Based on Improved GLR Algorithm

This article has been retracted.

**DOI:** 10.1155/2022/4105942

**Published:** 2022-04-15

**Authors:** Laiying Deng, Xinde Hu, Fen Liu

**Affiliations:** ^1^Guangzhou City Polytechnic, Guangzhou, Guangdong 510000, China; ^2^Beijing Qingneng Internet Technology Co., Ltd, Guangzhou Branch, Guangzhou, Guangdong 510000, China

## Abstract

Aiming at the problem of low accuracy of traditional algorithm model, an intelligent recognition model of business English translation based on an improved GLR algorithm is proposed. Through this algorithm, the automatic sentence recognition technology is established, and according to the characteristics of business English, the improved GLR algorithm is used for collection, sorting, and analysis, so as to realize the intelligent recognition of business English. The results show that based on the improved GLR algorithm, the recognition accuracy is high, and the comprehensive score is 92.5 points, which overcomes the disadvantages of the GLR algorithm, and the operation speed and processing are improved. Based on the improved GLR algorithm, the intelligent translation of business English is realized, which is accurate and fast, and greatly promotes the learning and development of business English.

## 1. Introduction

After joining the WTO, China's international business exchanges have become more frequent, the foreign trade industry has developed rapidly, and the demand for business English talents is increasing day by day. In this context, more and more colleges and universities begin to set up business English majors [1]. Business English translation course is an important skill course of this major, focusing on translation teaching. International business communication is mostly completed through language communication, and one of the common languages is English. The main communication language between Chinese businessmen and foreign countries is English. Therefore, the importance of business English translation teaching is self-evident. Recently, as the science and technology develop, the artificial intelligence is more and more widely applied, and machine translation is constantly updated and upgraded, which poses a challenge to the traditional human translation. There are some new problems in the teaching of business English translation in Colleges and universities, mainly manifested in the lagging consciousness of teachers, the outdated content of teaching materials and the single teaching methods [2–4].

As far as teachers' awareness is concerned, under the current situation that the functions of translation software are constantly upgraded and updated, many teachers do not understand the advantages and disadvantages of machine translation timely and fully. They can neither make use of its advantages in teaching nor face the challenges it brings, so as to adjust the teaching content accordingly [5]. As far as the content of teaching materials is concerned, although the quantity and quality of business English translation teaching materials on the market have improved in recent ten years, due to the limited factors such as long publishing cycle, limited energy of teachers, difficulty in collecting high-quality translation materials, rapid development of business society, the content of teaching materials cannot be updated in time, and the listed cases are relatively outdated. In terms of teaching methods, at present, in business English translation classes in colleges and universities, many teachers still use traditional teaching methods, focusing on theory, culture teaching, and translation practice. Sometimes, the explanation of translation theory is too much and too detailed. When arranging translation practice exercises, some translation examples are outdated, and the form and type of translation tasks tend to be single. Teachers' guidance of students' translation is not enough, so the effect of translation practice is not satisfactory, which affects the realization of the goal of talent training. It can be said that teaching methods have not been adjusted and improved according to the development, changes and trends of the times, society, and translation. In a word, the teaching of business English translation course cannot advance with the times, which is disconnected from the needs of society and industry. Therefore, there is an urgent need for reform in all aspects [6–8].

Machine translation, also known as automatic translation or computer translation, begins to develop in the 1940s. After years of development, it has gradually transformed from a very optimistic automatic high-quality machine translation to a more realistic and feasible computer-assisted translation. We can be seen the ideal of realizing unmanned translation was born as early as the 1940s, and CAT evolved from the original machine translation. During the development of computer-assisted translation, major business giants have also launched automatic translation services, such as Google translate and Baidu translate. In 2017, the artificial intelligence translation box appeared, and the speed and accuracy of the product's bilingual translation of everyday words are amazing. Instant artificial intelligence translation becomes a hot topic of discussion.

Recently, with the rapid development of intelligence, the use of computer technology to translate English has become the mainstream of the times. Now, there is a large market demand. Companies, universities, and professionals are like to use intelligent translation technology to translate business English, which brings great convenience and reveals that some machine translation levels have been unable to meet the current translation needs [9]. The market urgently needs a machine translation technology with high performance and high translation accuracy [10, 11]. The core idea of computer-aided translation is the translations are usually regarded as auxiliary references, so the users could obtain the advantages of translation and make manual selection. On the other hand, the use of corpus can classify and sort out the vocabulary in various industries, so that the quality of translation can be improved and closer to the actual needs of users. The rational use of professional vocabulary corpus with high translation frequency can not only greatly reduce repetition and translation workload but also greatly improve the accuracy of translation [12].

With the help of big data, the translation results of artificial intelligence translation software can be obtained instantaneously, which is conducive to learners' more efficient learning and consolidate their own learning effect [13, 14]. In other words, if they do not review after learning, the longer it takes, the less memory, or even forgetting. Learning needs to be reviewed constantly. By the artificial intelligence translation, we can learn faster and review better. No matter when and where we don't know, we can check if we are uncertain and review if we think of it. With the timeliness of the Internet, we can carry out more meaningful learning, reduce mechanical learning, and improve learning efficiency.

Students can use online cloud translation and online electronic dictionary to assist learning and make learning more efficient [15, 16]. Many students like to look at the word list and hold the word book to memorize words, but such learning is fragmented learning. They can only see the trees but not the forest. If they remember the words, they may not be able to use them. Learning is easy to be frustrated. However, the use of intelligent translation-assisted learning can avoid the situation of learning words without understanding the application and can get through the vocabulary more quickly and better, because intelligent translation presents learners with complete sentences rather than fragmented language. We can even make use of the advantage of intelligent translation based on big data to select corpus closer to our lives and our favorite fields for learning, so as to make learning more interesting and grounded. This is especially suitable for students with a slightly poor foundation. They can use translation software to make up for the personalized needs that cannot be met in the big classroom, improve their interest in learning, make up for their shortcomings, and make learning happen continuously.

Under the influence of the Internet and big data, the language learning model needs to be changed [17]. Foreign language learners can no longer be limited to the learning of words, phrases, and simple sentence patterns but should develop more comprehensive abilities. Compared with the past, using the mobile app to assist learning, improving listening, or writing ability by visiting web pages, and using the fragmented time to read English novels to improve reading ability, intelligent translation is more comprehensive and effective in assisting learning [18]. Students can not only master the grammar and grammar but also improve their ability to translate and use the words intelligently.

Zhou [19] analyzed the detailed features of machine translation in Business English, adopted the NT clause as the unit in English translation, and then achieved the purpose of business English translation through the PTA model, which reflected the intelligence of small languages. Lu [20] improves the traditional intelligent recognition model of business English translation and adopts the language intelligent translation model. Firstly, the sinusoidal similarity algorithm is used to obtain the measurement values of different semantics, so as to obtain the accuracy of business English translation and ensure the accuracy of business English. Huang [21] used the analytic hierarchy process to analyze the business English translation and made a sentence comparative analysis of the English Thesaurus and the cut words, so as to obtain the possible grammatical composition of business English, reduce the error rate of business English translation, and improve the accuracy and accuracy of the translation.

In general, this paper implements a sentence tagging system suitable for small and medium-sized syntactic tagging corpus method analyzers. In the implementation process, in order to improve the sensitivity of lexical annotation information to differences, the number of rules shall be reduced as far as possible, and the text shall be marked at the first level, but the verbs shall be marked. At the same time, some auxiliary words and punctuation in sentences are labeled in detail, so that some ambiguities can be eliminated through detailed part of speech labeling information in the ruling stage [22]. Structural ambiguity is a difficulty in the field of English translation, which needs to be solved by part of speech recognition algorithm. In order to use English in daily communication practice, we should strengthen English pronunciation correction and learning. In the past, it was completely taught by teachers, which not only required a lot of human resources but also difficult to realize. Therefore, it is particularly important to develop an intelligent recognition model for English translation. The model can monitor students' English pronunciation and put forward correction suggestions. There are some problems in the traditional intelligent recognition model and setting of the English translation, which cannot accurately recognize English translation and cannot correct students' English pronunciation, but also mislead students' pronunciation and affect English learning.

Based on the above problems, this paper establishes a language database, improves and analyzes the GLR algorithm, establishes an improved GLR algorithm model, and achieves the function of intelligent recognition. According to the syntactic function of parsing the linear table, this paper corrects the English Chinese structural ambiguity in the part of speech recognition results, finally obtains the recognized content, and determines the actual position range of phrases in translation, in order to alleviate the disadvantages of structural ambiguity in the current field of the English translation to a certain extent and to improve the efficiency of phrase recognition. Finally, an intelligent recognition model of business English translation based on an improved GLR algorithm is established to automatically recognize English translation. In order to verify the effectiveness of the model, simulation experiments are carried out in the simulation environment.

## 2. English Intelligent Recognition Algorithm

### 2.1. Creating Phrase Corpus

In Chinese, words are divided into notional words and functional words. Notional words refer to those components that express real meaning, can be used as phrases or sentences, and can form sentences alone. Function words generally do not express real meaning and are not used as components of phrases or sentences (except adverbs). Their basic purpose is to express grammatical relationships. In order to obtain as many analysis results as possible, thread technology is adopted to display all the possible analysis results of one sentence for the probability model to choose the best one [23].  Figure 1 shows the information flow of the phrase corpus.

The English translation intelligent recognition model designed in this paper has more than 500000 words in the phrase corpus, which can meet the needs of practical use. As shown in Figure 1, the phrase corpus is highly targeted. Through the English Chinese machine translation phrase corpus, this paper comprehensively distinguishes the tenses of different phrase corpora and labels the English Chinese phrase corpus. The corpus marking method includes three parts: level, data, and processing. The data type is text format. The level uses alignment and part of speech.

### 2.2. Phrase Corpus Part of Speech Recognition

Noun phrase is a very important phrase type, which accounts for a large proportion in Chinese sentences. Recognizing short nouns is a very important subtask in the field of natural language processing. It is directly related to the correctness of text analysis and text processing. As a preprocessing method of natural language processing, its analysis results can simplify the sentence structure and solve the ambiguity problem, so as to reduce the difficulty and complexity of syntactic analysis and provide the basis for further phrase division and syntactic analysis. At the same time, it is of great significance to the application fields of machine translation, information retrieval, information extraction, and corpus research [24].

GLR algorithm, also known as the Futian algorithm, is an extended LR algorithm. The algorithm introduces graph structure stack, subtree sharing, and local ambiguity reduction. In order to make the space complexity as small as possible in the process of constructing the item set family of the algorithm, the merging strategy of item set is adopted; In order to obtain as many analysis results as possible, thread technology is adopted to display all the possible analysis results of one sentence for the probability model to choose the best one.

The operation of each step of the classical GLR algorithm uses a variety of shift instructions and simplified operations. The beginning and terminal of each operation during the period are displayed using the special envoy's standard. In the process of phrase translation, when the GLR algorithm does not detect grammatical ambiguity, it will restart the operation of deduplication and calibration. If grammatical ambiguity is detected, it is necessary to use the geometric structure linear table of syntactic analysis, which provides the optimal content according to the local optimization principle, transports it to different recognition channels for symbol recognition, and selects the optimal result according to the recognition result [25].

Generally, the traditional GLR algorithm has a low degree of character recognition, so it cannot effectively translate business English and apply more accurate English translation. Based on the improved GLR algorithm, this paper establishes the automatic recognition ability, which greatly improves the accuracy of sentence recognition as shown as follows:

(1) $$\begin{array}{c} G_{E}\;=\;\left(V_{N},V_{T},S,\alpha \right). \end{array}$$

If *P* represents *α* any action in and exists in *V*_*N*_, such as language translation, grammar checking, speech recognition, and other actions. Through derivation, it can be concluded that

(2) $$\begin{array}{c} \text{P}⟶\left\{\theta \text{,c,x,}\delta \right\}. \end{array}$$

When doing the GLR based parsing algorithm, due to the splitting of some concentric sets in the process of constructing the state transition graph, the number of result states increases sharply, resulting in a sharp increase in the complexity of program space and a large amount of memory space. When there are many rules, the execution of the program will overflow the memory [26].

## 3. English Translation Intelligent Recognition Model

The intelligent recognition model is planned according to data collection, processing, and output.  Figure 2 shows the overall architecture of intelligent recognition of business English translation.

### 3.1. Model Design Process

The functions are planned required by the English translation intelligent recognition model, and the overall model is designed.  Figure 3 shows the model design process. This model can realize data collection, output, and processing. The data acquisition device is used to collect the voice signal, and then, the audio input device is used to input the English signal into the processing system to process the data signal. The processed results are output in the corresponding client and displayed. The user can view the automatic recognition results of English translation through the display or client.

### 3.2. English Signal Processing

After the model design, we should carry out a detailed design, collect, and process English signals in a planned way. However, because English speech signals have interference factors, such as nonstandard pronunciation of the human body and imperfect equipment, the collected speech signal information is not 100% accurate. In order to improve the accuracy, the collected voice signals should be processed, including framing, weighting, endpoint monitoring, and windowing.

The digital filter is used to realize the speech signal weighting processing and improve the stress detection system. The specific method is to use the symbols *F*1 and *F*2 to represent the first and second formants of vowel spectrum characteristics, respectively, which are related to the front and back of tongue position and high and low. Based on this, after using a neural network to distinguish nonstress and stress, we can use the classifier system to output position confidence, so as to measure the vowel intonation, and then select the best speech signal. In this paper, the high-frequency signal lifting pre-emphasis digital filter with a signal-to-noise ratio of 6 dB is used to process the frequency band of speech signal higher than 800 Hz. Weighting coefficient *α* between 0.9 and 1.0, the calculation formula of weighting processing signal *y* (*n*) is

(3) $$\begin{array}{c} y\left(n\right)=T\left[x\left(n\right)\right]=ax\left(n\right)+b\left(a\;\mathrm{and}\;b\text{ are constants and not 0}\right)\text{,} \end{array}$$

where *x*(*n*) is the input voice signal. Among them, a can be taken according to the high-frequency signal, and *b* is the frequency band value, which can be obtained according to the experimental results. After signal processing, the voice signal is processed in the second step, and the half-frame overlapping method is used to realize the framing operation. In order to accurately analyze the speech signal, the speech signal is divided into *t* frames, and the calculation formula is

(4) $$\begin{array}{c} z\left(n\right)=\frac{1}{t}y\left(n\right), \end{array}$$

where *z*(*n*) is the speech signal after dividing the *t* frame. After the framing operation processing is realized, the voice signal is windowed. In order to clearly show the voice effect, the rectangular window *w*(*n*) is selected, and the calculation formula is

(5) $$\begin{array}{c} w\left(n\right)=\omega \left(n\right)\times z\left(n\right). \end{array}$$

*ω*(*n*) is the windowed speech signal, which has a fast response and improves the translation accuracy. The endpoint monitoring of processed speech signal is realized by using the double threshold comparison method, so as to quickly find the starting point and ending point for data processing and storage. This method can reduce the interference items and improve the monitoring accuracy.

### 3.3. Extracting Characteristic Parameters

In order to train the later feature extraction and parameter estimation, the corpus must be preprocessed first. Each word is extracted in the text and its context information to form a word item, and the frequency of the same word item is recorded. All word items form a thesaurus containing all the characteristic attributes of each word and its context.

In the test model, the input text is preprocessed to obtain the feature information of each word and its context, and then, the feature vector satisfied by the word is calculated; finally, the feature vector and feature parameters are used to label the right part of the feature, and the maximum labeling result is the final labeling result. Through the improvement of a finite length discrete speech signal, the following formula is obtained:

(6) $$\begin{array}{c} X\left[K\right]=\sum_{n=0}^{N-1}x\left[n\right]e^{-j\frac{2\pi }{N}\;nk},k=0,1,2,...,N, \end{array}$$

where *x*[*n*] is the discrete speech sequence obtained by sampling, and *X*[*K*] is the *k*-point reset sequence.

Discrete speech sequences are transformed into Mel frequency scales.

(7) $$\begin{array}{c} \mathrm{Mel}\left(f\right)=2579\mathrm{lg}\left(1+\;\frac{f}{700}\right), \end{array}$$

where Mel (*f*) is the Mel frequency and *f* is the actual frequency.

Discrete cosine transform DTC on the filtered output is carried out to obtain the feature parameter extraction result *P* of speech signal *w*(*n*). The calculation formula is

(8) $$\begin{array}{c} P=Z_{n=1}^{N}F\left(l\right)w\left(n\right)\cos\left(\pi n\left(M+0.5\right)\right). \end{array}$$

When an improved GLR algorithm is used to analyze sentences, it will first reduce the complexity of sentences and then adopt automatic recognition technology to translate business English through the function of its own algorithm. Moreover, under the intelligent recognition technology, using the above method, taking English speech intelligent recognition as the demand, the relevant speech signal parameters are extracted from the aspects of rhythm, speed, intonation, and intonation.

## 4. Test and Model Verification

### 4.1. Verification Scheme

In order to verify the actual English Chinese translation effect of the improved GLR algorithm, based on the above methods, this paper preliminarily realizes a prototype system and preliminarily carries out some experiments for the word alignment method based on dictionary and semantic similarity, the word alignment method based on statistics, and the method based on the integration of statistics and dictionary to test the effectiveness of different word alignment methods. The influence of noun phrase alignment based on word alignment position information is proposed in this paper. Afterwards, the dictionary-based method combines the advantages of the statistical method and the dictionary-based method, which not only makes up for the lack of accuracy in the statistical method, increases the number of correct alignment, and ensures the accuracy of nonempty alignment but also overcomes the problem of limited dictionary coverage in the dictionary-based method, and further improves the translation accuracy of business English.

### 4.2. Experimental Results

Through the intelligent recognition technology of business English, the results are shown in Figure 4. It can be seen that the improved GLR algorithm for part of speech recognition is the best in the same category, followed by the GLR algorithm, and the worst is the statistical algorithm. From Figure 5, we can find that the improved GLR algorithm can obtain the high score, which is 92.5 points, and the statistical algorithm is 76.0 points, which is the lowest.  Figure 6 shows the frequency intensity analysis under different algorithms. It can be seen that the frequency intensity of the improved GLR algorithm is relatively stable and close, while the intensity of the statistical algorithm under different frequencies is poor, which shows that the translation accuracy of the improved GLR algorithm is the highest. In general, machine translation based on the statistical algorithm and dynamic memory algorithm did not translate the word “Price Bureau,” but machine translation based on improved GLR algorithm correctly translated it. When translating the “explanation,” only the machine translation based on the improved GLR algorithm is closest to the human translation. It can be seen that the machine translation based on the improved GLR algorithm designed in this paper is more accurate than the statistical algorithm and the dynamic memory algorithm, reaching the same level as the human translation. Chinese Grammar presents integrity, fuzziness, and high flexibility; English grammar is highly systematic. Due to the limited vocabulary of learners, their understanding of language knowledge is not comprehensive. The mastery of grammar rules is ambiguous and limited by the Chinese way of thinking. Their foreign language learning generally has a thinking transformation process from English to Chinese and then to English. This kind of error is almost difficult for learners to detect without teachers' guidance, so teachers should point out and correct this kind of error. It shows that the improved GLR algorithm is efficient and feasible in machine translation. Combined with Figures 4to 6, the improved GLR algorithm has a higher score and better intelligent pattern recognition.

Figure 7 shows the distribution of section control points identified by the system. It can be seen that the syntax and phrase recognition system obtained by the statistical algorithm has loose node distribution, while the syntax and phrase obtained by the dynamic memory algorithm and GLR algorithm have a compact node distribution, indicating that the intelligent recognition technology of the representation model is high and the translation accuracy is good. The compact distribution of node control points obtained by the improved GLR algorithm shows that the system is easy to operate and has high precision, which is helpful for business people to use, and can promote the rapid development of business English translation.

Each algorithm has its unique advantages. In this paper, the applicable places of various algorithms are discussed in detail and then applied to the teaching management of business English. Its advantages and disadvantages are compared, so as to better highlight the advantages of an improved GLR algorithm.  Figure 8 shows the proportion of different algorithms in Business English translation. It suggests that the improved GLR algorithm is the most widely used, accounting for 40%, followed by the GLR algorithm, and the statistical algorithm is the lowest, accounting for only 10%. This shows that the improved GLR algorithm is the most commonly used in Business English translation, which is consistent with the above analysis results. The application potential of the improved GLR algorithm in Business English intelligent translation is unlimited. For business English in high-frequency compound noun phrases, many statistical indicators can be obtained effectively. For low-frequency compound noun phrases, less language phenomena can be observed in the corpus, and various statistical indicators do not perform well. Therefore, based on the improved GLR algorithm, high-frequency compound noun phrases are used to help find low-frequency compound noun phrases, so as to achieve the results of intelligent automatic translation of business English.

## 5. Conclusion

Aiming at the structural problems existing in English translation, an improved GLR algorithm is proposed to solve the data point coincidence problem in the traditional GLR algorithm. The phrase structure in the improved algorithm is designed by using the phrase center point to analyze the syntactic function of the linear table, correct the ambiguity of part of speech recognition structure and English Chinese structure, solve the problem of low accuracy of recognition results in traditional calculation methods, and provide a reasonable method for phrase recognition. The experimental results show that compared with other algorithms, the machine translation based on the improved GLR algorithm has the characteristics of simple and fast calculation, low difficulty, and stronger practicability. In general, the improved GLR algorithm meets the needs of English machine translation and is suitable for English machine translation.

## Figures and Tables

**Figure 1:** Phrase corpus information flow.

**Figure 2:** General framework of intelligent recognition of business English translation.

**Figure 3:** Model design process.

**Figure 4:** Evaluation results of four English Chinese translation algorithms.

**Figure 5:** Comparison of comprehensive test scores of four English Chinese translation algorithms.

**Figure 6:** Frequency intensity analysis under different algorithms.

**Figure 7:** The distribution of control points of the system.

**Figure 8:** Proportion of different algorithms in business English translation.

## Data Availability

No data were used.
